# Hydroxyethyl Starch Improves the Prognosis of Rats with Traumatic Shock via Activation of the ERK Signaling Pathway in Lymphocytes

**DOI:** 10.1155/2022/5262189

**Published:** 2022-02-08

**Authors:** Yun Liu, Jian Lu, Caifu Dong, Limin Zhu, Li Zhou, Kai Zhu

**Affiliations:** Department of General Surgery, Ningbo Zhenhai Longsai Hospital, Ningbo, Zhejiang Province 315200, China

## Abstract

**Objective:**

Severe traumatic shock is one of the leading causes of death in young adults. A large number of studies have shown that effective volumetry resuscitation on the basis of controlled injury can not only increase the success rate of early resuscitation but also reduce systemic inflammatory response and improve the cure rate of severe traumatic shock. The study explored the effects of hydroxyethyl starch (HES) on the survival rate, lymphocyte function and proliferation of rats with traumatic shock, and the potential mechanisms.

**Methods:**

Traumatic shock was constructed in rats as experimental model, and liquid resuscitation was performed using HES and lactated Ringer's (LR). 24-h mortality was recorded, and lymphocytes were isolated. The expressions of signaling pathway factors was detected by qPCR and Western blot. ELISA was performed to determine the expression of interleukin 6 (IL-6) and tumor necrosis factor-*α* (TNF-*α*) in cell supernatant.

**Results:**

HES for fluid resuscitation augmented the survival of traumatic shock rats, upregulated the expressions of MEK and ERK1/2, and downregulated the expressions of IL-6 and TNF-*α*. However, inhibition of ERK signaling pathway reversed the effect of HES on the immune improvement and the 24-h survival rate of the traumatic shock rats (*P* < 0.05).

**Conclusion:**

HES could exert the anti-inflammatory effects on lymphocytes by mediating the phosphorylation of proteins of the ERK signaling pathway. HSE demonstrated a high efficacy in effectively treating traumatic shock, thus could be used in clinical practice.

## 1. Introduction

Severe trauma is often accompanied by a large amount of blood loss. Multiple organ failure, severe systemic reactions, and even death could occur as a result of insufficient blood and oxygen supply to local tissues. Traumatic shock has therefore become the main cause of death within 24 hours (h) after admission to hospital, and it accounts for more than 9% of the global mortality [1, 2]. However, death as such can be prevented by prompt and effective medical measures. Timely replenishment of body fluids can help prevent complications such as dehydration and renal failure. Hydroxyethyl starch (HES) and Ringer's lactic acid (LR), which are two different colloids widely used in fluid resuscitation, can effectively improve the prognosis of patients with traumatic shock under point-of-care application [3]. Hydroxyethyl starch can “block” capillary leakage, effectively improve the hemorheological abnormalities of microcirculation, and increase tissue oxygen supply [4]. HES can significantly reduce the systemic inflammatory response and vascular endothelial injury after traumatic shock [5]. At the same time, it may induce the changes of lymphocyte proliferation and differentiation by destroying the balance of proinflammatory response and anti-inflammatory response marked by the level of serum IL-2, IL-4, *γ*-IFN, etc. [6].

As a major mechanism of trauma stress, the inflammatory response not only plays an important role in activating the immune system and resisting infection, but also induces cytokine storms that can lead to tissue and cell damages and/or even multiple organ failure, thereby greatly contributing to the poor long-term life quality of patients survived from traumatic shock [7]. The changes of lymphocytes after trauma include changes in quantity and function. Bone marrow suppression, thymus paralysis, and the decrease in the number of peripheral blood lymphocytes are common after severe trauma. The number of CD4+ and CD8+ cells decreases, especially the number of CD4+ cells, which leads to the decrease or even inversion of the ratio of CD4+/CD8+, resulting in the decline of the function of producing lymphokines, assisting cells to produce antibodies and assisting other lymphocytes. At molecular level, the expressions of interleukin 6 (IL-6) and tumor necrosis factor-*α* (TNF-*α*) are often upregulated in body's inflammatory responses including in cell growth and differentiation, and the two serve as the most common circulating markers indicative of inflammatory response [8]. As an important protein kinase in MAPK signal transduction, ERK regulates a variety of cellular activities including cell proliferation and survival [9]. Moreover, PI3K and its downstream mediators Akt and mTOR are closely involved molecules in cell survival, proliferation, and metabolism [10]. Therefore, molecules related to lymphocyte proliferation may play a critical role in the damage of organism caused by traumatic shock. After traumatic shock, the differentiation and proliferation of lymphocytes changed significantly. Early hydroxyethyl starch resuscitation may avoid this trend and protect body's immunity.

Studies discovered that low-dose HES and LR used for fluid resuscitation has a remarkable effect that can better maintain homeostasis, hence significantly improve the survival rate of patients [11]. Moreover, HES can greatly alleviate the proinflammatory response and immunosuppression that may occur in surgical operations [12]. Thus, we hypothesized that the fluid resuscitation using HES may be related to lymphocyte apoptosis. The novelty and motivation of this study is to investigate whether the fluid resuscitation using HES is related to lymphocyte apoptosis and detect the relationship between HES and ERK signaling pathway for the first time. In this study, the rat model of traumatic shock was constructed to explore the effect of HES resuscitation on lymphocytes in traumatic shock rats and the potential molecular mechanism.

## 2. Materials and Methods

### 2.1. Experimental Animals

We purchased 210 SPF-grade SD male rats (9-11 weeks old, weighing 250-300 g) from Beijing Viton Lihua Laboratory Animal Co., Ltd. (production license SCXK, Beijing, 2016-0006). The rats were divided into following 7 groups according to the random number table, 30 rats of each group: sham group (sham operation group), HES group (HES resuscitation group), LR group (LR resuscitation group), CON group (trauma control group), U0126 + HES group (mixture of ERK1/2 inhibitor U0126 and HES recovery), LY294002 + HES group (mixture of PI3K/Akt inhibitor LY294002 and HES recovery), and U0126 + LY294002 + HES group (mixture of ERK1/2 inhibitor U0126, PI3K/Akt inhibitor LY294002 and HES recovery). All the rats were fed for 1 week for adaptation prior to the experiment. This experiment was approved by the Animal Ethics Committee of Ningbo Zhenhai Longsai Hospital and performed strictly according to NIH Guide for the Care and Use of Laboratory Animals [13].

### 2.2. Experimental Method

#### 2.2.1. Construction of Rat Model

One week before modeling traumatic shock, the rats in U0126 + HES group, LY294002 + HES group, U0126 + LY294002 + HES group, and CON group were, respectively, administrated with U0126 (Invivogen, tlrl-u0126, 0.1 mg/kg), LY294002 (Invivogen, tlrl-ly29, 0.3 mg/kg), and U0126 + LY294002 (0.1 mg/kg+0.3 mg/kg) and intraperitoneally injected with normal saline of same amount (once a day for 7 days in total).

The rats were anesthetized by intraperitoneally injecting 1% pentobarbital sodium (40 mg/kg, Shanghai Xinya Pharmaceutical Co., Ltd., H31021725), the left femoral artery was separated from femoral vein, and the pressure transducer was connected to the femoral artery. Real-time blood pressure was monitored, and the femoral vein was cannulated for resuscitation. Traumatic fracture of the right femur was established on the rats, and blood was drawn from the left femoral artery. If MAP continued to drop, lactated Ringer's solution was infused via the jugular vein cannula to maintain a 35-mmHg MAP. In some rats, traumatic injury was not severe enough to lower MAP to 35 mmHg. In some rats, the traumatic injury was not serious enough to reduce the MAP to 35 mmHg; thus, a heparinized catheter was placed in the left femoral artery, and blood was drawn until the map decreased to 35 mmHg in these rats. The model of traumatic shock was considered successful when the average arterial pressure (MAP) was reduced to 35~40 mmHg and maintained for 1 h. Subsequently, fluid resuscitation was performed immediately [14].

The rats of HES group, U0126+HES group, LY294002 + HES group, and U0126 + LY294002 + HES group were intravenously injected with 6% HES130/0.4 (Huaren Pharmaceutical (Rizhao) Co., Ltd., H20061095, 20 ml/kg ∗ h); the rats in the LR group were injected with LR (Luan Huayuan Pharmaceutical Co., Ltd., H20033520, 20 ml/kg ∗ h); the rats in the CON group were injected with saline (Beijing Tiantan Biological Products Co., Ltd., S10870001, 20 ml/kg ∗ h). Hemorrhage was performed 1 h after the corresponding injection, and fresh whole blood was infused into the rats. The resuscitation was considered as completed after MAP reached 80 mmHg and HCT reached 30% and maintained for more than 1 h. No other operations were performed in the sham group except for femoral artery and venipuncture catheters.

After resuscitation, the vein cannula was removed, femoral vein was ligated to stop bleeding, wound was closed, and antibiotics were intramuscularly injected to prevent infection. The rats were fed with normal diet, their survival and time of death of rats were recorded, and the 24-h survival rate was calculated. All the rats were sacrificed by neck dislocation after 24 h of recovery.

#### 2.2.2. Preparation of Lymphocyte Suspension and Lymphocyte Culture

The sacrificed rats were immersed in 75% alcohol and placed on a benchtop. Spleens of rats were removed, and the connective tissues were cleared away. Then, the spleens were rinsed in PBS, minced by ophthalmic scissors, and grinded into cell suspension using pestle. The cell suspension was then rinsed in DMEM medium and were transferred into Percoll (Sigma, P1644) and centrifuged at 1000 rpm for 10 min in a centrifugal tube, then spleen lymphocytes were isolated from the Percoll gradient separation interphase. Red blood cells were lysed for 5 min by red blood cell lysis buffer (Solarbio, R1010) and washed by centrifuging at 1000 rpm for 5 min. Next, the supernatant was discarded, and the cells were resuspended. Part of the resuspended cells was cultured in RPMI-1640 (Gibco, 61870036) medium containing 10% FBS (Gibco, DXT-10099141), while the rest was washed, diluted by PBS, and fixed by ethanol.

#### 2.2.3. Detection of IL-6 and TNF-*α* in Lymphocyte Culture Medium Using ELISA

After incubation for 24 h, the cell culture medium was centrifuged at 1000 rpm for 10 min to obtain the supernatant for the assay. With standard wells and sample wells setout, 50 *μ*l standards of different concentration were added to the standard wells, 10 *μ*l samples and 40 *μ*l diluent were added to the sample wells to be tested, 100 *μ*l HRP-labeled antibody diluent was added to each well except the blank wells, then the reaction wells were sealed and incubated at room temperature for 1 h. The supernatant was discarded and the wells were washed 5 times. Substrate solutions A and B were added in sequence and incubated for 15 min in the dark. Subsequently, 50 *μ*l stop solution was added into each well, and the OD value at 450 nm was measured using an automatic microplate reader (Biorad, iMark) within 15 min. ELISA kits for IL-6 and TNF-*α* were purchased from Abcam company (article numbers ab234570 and ab100785).

#### 2.2.4. QPCR Detection

Trizol (Gibco, DXT-15596018) was used to extract total RNAs from lymphocytes, RNA reverse transcription was performed according to the instructions of the kit (Thermo, BTK1622), and the cDNA library was prepared after dilution. The target sequence was amplified by a fluorescent quantitative PCR instrument (ABI, 7500). The primer sequences were designed and synthesized by Shanghai Gema Co., Ltd. (see Table 1 for details).

For the reaction system, 2 *μ*l cDNA, 0.6 *μ*l forward and 0.6 *μ*l reverse primers, 10 *μ*l FastFire qPCR PreMix (Tiangen Biochemical Technology (Beijing), FP208-01), and RNase-Free ddH2O were mixed thoroughly for a 20 *μ*l reaction system.

The amplification procedure conditions were set as follows: predenaturation at 95°C for 1 min, followed by denaturation at 95°C for 5 sec, annealing/extension at 55°C for 15 sec, for a total of 40 cycles. 3 duplicated wells for each group were set up, and the relative expression of the target gene was calculated using 2^−△△^Ct method.

#### 2.2.5. Detection of Protein Expression Using Western Blot

The total proteins from lymphocytes were isolated by RIPA (Biorbyt, orb402072) protein lysate, separated by 10% SDS-PAGE gel electrophoresis, and transferred onto a membrane for 90 min. Then, the membrane was blocked at room temperature for 1 h using 1% BSA (Solarbio, PC0001), primary antibody dilutions MEK (Abcam, ab32091), ERK1/2 (Abcam, ab17942), p-MEK (Abcam, ab96379), p-ERK1 (Abcam, ab200807), p-ERK2 (Abcam, ab151549), PI3K (Abcam, ab106693), Akt (Abcam, ab2732), mTOR (Abcam, ab182651), p-Akt (Abcam, ab192623), p-mTOR (Abcam, ab137133), and *β*-actin (Abcam, ab8227) were subsequently added and incubated at room temperature for 2 h. After washing the membrane three times with TBST buffer, the cells were added with HRP-labeled secondary antibody (Abcam, ab205718) and incubated at room temperature for 0.5 h, then washed with TBST buffer for three times. The protein bands were developed by ECL luminescence kit (Absin, abs920) for detection.

### 2.3. Statistical Analysis

All in vitro assays were conducted for three biological and technical replicates. The data were calculated and plotted using GraphPad 8 and shown as (mean ± sd). Independent-sample *T* test was in comparison of two groups, while one-way ANOVA was used in comparison among multiple groups, LSD-t was used for post hoc test. *P* < 0.05 were considered as statistically significant.

## 3. Results

### 3.1. HES Resuscitation Improved the Survival Rate of Traumatic Shock Rats

After resuscitation, all rats in the U0126 + LY294002 + HES group died within 24 h. The mortality rates of the HES group, LR group, CON group, U0126 + HES group, and LY294002 + HES group were 10%, 16.67%, 66.67%, 43.33%, and 40%, respectively, while no death occurred in the sham group within 24 h. As shown in Figure 1, the Kaplan-Meier method was used to plot the 24 h survival curves of traumatic shock rats in each group. The 24 h survival rate of the sham, HES, LR, CON, U0126+HES, LY294002+HES, and U0126+LY294002+HES group was 100%, 90%, 83.33%, 40%, 60%, 60%, and 0%, respectively, and the survival rate of the HES and LR group was significantly higher that of CON, U0126 + HES, LY294002 + HES, and U0126 + LY294002 + HES group (*P* < 0.05). HES and LR resuscitation could reduce the 24 h mortality rate of traumatic shock rats, whereas the administration of pathway inhibitors U0126 and LY294002 could attenuate the curative effect of resuscitation using HES (*P* < 0.05).

### 3.2. HES Affected Lymphocyte Proliferation and Inflammation

The results of flow cytometry showed that the apoptosis rate of lymphocytes in LR and CON groups was significantly higher than that in sham and HES groups (*P* < 0.05). QPCR and Western blot analysis demonstrated that the expression levels of MEK1, p-MEK, and p-ERK1/2 were greatly higher in HES groups than those in sham, LR, and CON groups (*P* < 0.05). In addition, ELISA was used to detect the expression levels of IL-6 and TNF-*α* in cell supernatants, and we found that the CON group showed higher expression levels than sham, HES, and LR groups and that the LR group had higher expressions than the sham group (*P* < 0.05). However, as shown in Figure 2, no significant difference was found in the expressions of inflammatory factors between the HES and sham groups (*P* > 0.05).

### 3.3. Inhibition of ERK Signaling Pathway Reversed the Antiapoptotic Effect of HES on Lymphocyte

The results of flow cytometry showed that the apoptosis rate of lymphocytes in U0126+HES and U0126+LY294002+HES group was higher than that in HES group (*P* < 0.05); there was no significant difference in apoptosis rate between LY294002+HES group and HES group (*P* < 0.05). QPCR and Western blot analysis showed that U0126 significantly inhibited the protein expressions of p-MEK and p-ERK1/2 in U0126+HES groups than in HES groups and that LY294002 greatly inhibited the protein expressions of p-MEK, p-ERK1/2, p-Akt, and p-mTOR in LY294002+HES groups than HES groups (*P* < 0.05). However, U0126 was found to noticeably reverse the downregulatory effect of HES on the expression levels of IL-6 and TNF-*α* in the lymphocyte supernatant (*P* < 0.05) (as shown in Figure 3).

## 4. Discussion

ERK is a typical signaling pathway of cell proliferation, and it can exert antiapoptotic effect on various cells. ERK protein can be activated by phosphorylation and subsequently translocated into the nucleus to regulate the activity of the transcription initiation sites (such as cAMP response element binding proteins) that are associated with cell survival [15], thereby improving cell survival. Studies showed that ERK and its upstream kinases, MEK, MAP, etc., play critical roles in the regulation of immune cell functions via regulating immune system signals, acute inflammation, etc. [16]. The number of lymphocytes, which can reflect changes occurred in the blood and spleens, is indicative of the degree of hyperacute immune response during wound formation [7]. In this study, we discovered that compared with LR, fluid resuscitation of HES is significantly increasing the phosphorylation of MEK and ERK1/2 proteins in cells, while the proliferation effect of HES on lymphocytes was severely affected after using ERK signaling pathway inhibitor U0126. In addition, it has been previously discovered that inhibiting the phosphorylation of ERK protein greatly affects the proliferation of lymphocytes, bringing damage to the spleen of rats [7], which confirms our findings.

The prognostic survival of the traumatic shock rats was remarkably improved after fluid resuscitation using HES, which is consistent with previous studies [11, 17]. It should be noted that in their SD rat models of traumatic hemorrhagic shock, Masoumi et al. [18] discovered that HES resuscitation regulates the balance of TH1/TH2 response, inhibits NF-*κ*B activation, and promotes CD4+T cell apoptosis of the traumatic hemorrhagic rats, thus improving the immunosuppression, disorder, and inflammation of the rats, which is also in line with our results. In our study, the results of flow cytometry showed that the apoptosis rate of lymphocytes in LR and CON groups was significantly higher than that in sham and HES groups. In addition, the CON group showed higher expression levels than sham, HES, and LR groups and that the LR group had higher expressions than the sham group.

In acute inflammation, the activation of leukocytes often occurs after glycocalyx shedding, and it has been found that the resuscitation of colloidal fluids will further accelerate glycocalyx shedding, thereby exacerbating the inflammatory reaction [19]. However, a recent study showed that [20] HES can prevent the degradation and rupture of glycocalyx through reducing the plasma concentration of syndecan-1, thereby maintaining the integrity of vascular epithelium, preventing plasma leakage, and repairing vascular microenvironment damage caused by inflammation. HES shows a more rapid curative effect compared with LR and can better maintain blood pressure and provide adequate tissue oxygenation and peripheral perfusion in fluid resuscitation [21, 22]. Moreover, the nephrotoxic effect of HES [20] mainly manifests in patients with septic shock rather than those with hemorrhagic shock [23]. On the other hand, Li et al. [24] demonstrated that under inflammatory conditions, HES has an anti-inflammatory function through reducing neutrophil activation, platelet-neutrophil aggregation, and extraneutrophil trap. The current findings revealed that HES can effectively reduce the relative expressions of IL-6 and TNF-*α* in the cell supernatant. IL-6 serves as an important inflammatory signaling molecule, and its relative expression generally corresponds to immune response and the degree of tissue injury; thus, IL-6 is considered as an indicator for prognostic evaluation of patients with traumatic shock [25]. Tumor necrosis factor can mediate a complex signal regulation mechanism in traumatic shock, trigger body inflammation and cytokine storm, and even cause dysfunction of multiple organs including the heart [26]. Low-expressed IL-6 and TNF-*α* in lymphocytes after HES resuscitation indicate that HES can exert anti-inflammatory effects on traumatic shock rats.

The current experiment failed to demonstrate the effect of liquid resuscitation using concentration gradient of HES and LR together on traumatic shock, but 6% HES130/0.4 still showed significant resuscitation effect and anti-inflammatory effect on traumatic shock rats. In-depth study is required to further investigate the specific mechanism underlying the proliferation effect of HES on lymphocytes, which will be the direction of our future research.

In conclusion, using HES for fluid resuscitation can significantly improve the prognosis of traumatic shock rats and downregulate the expressions of IL-6 and TNF-*α* through the activation of phosphorylation of the ERK signaling pathway protein. Furthermore, HES can also serve as a significant fluid supplement to plasma in clinical resuscitation.

## Figures and Tables

**Figure 1:** Survival of traumatic shock rats in each group at 24 h.

**Figure 2:** HES attenuated lymphocyte apoptosis and inflammation. (a) Lymphocyte apoptosis rate; (b) QPCR was used to detect the relative expressions of various mRNAs in lymphocytes; (c) Western blot was used to detect the expression of lymphocyte protein; (d) ELISA was used to detect the expression levels of various inflammatory factors in the cell supernatant. ^∗^*P* < 0.05 vs. sham group; ^#^*P* < 0.05 vs. HES group; ^&^*P* < 0.05 vs. CON group.

**Figure 3:** The effect of inhibiting ERK signaling pathway on lymphocytes. (a) Lymphocyte apoptosis rate; (b) QPCR was used to detect the relative expression level of each mRNA in lymphocytes; (c) Western blot was used to detect the expression level of lymphocyte protein; (d) ELISA was used to detect the expression levels of various inflammatory factors in the cell supernatant. ^∗^*P* < 0.05 vs. HES group; ^#^*P* < 0.05 vs. U0126+HES group; ^&^*P* < 0.05 vs. LY294002+HES group.

**Table 1:** Primer sequence.

Primer		Primer sequence
ERK1	Forward	5′-AACTACCTACAGTCTCTGCCCTCT-3′
	Reverse	5′-GTGAGCCAGTGCTTCCTCTACT-3′
ERK2	Forward	5′-GCTGAATCACATCCTGGGTA-3′
	Reverse	5′-CTGTTCCACGGGCACCTTATT-3′
MEK1	Forward	5′-TGAGCCTCCTCCAAAACTGC-3′
	Reverse	5′-CCCCAAGCACAAAGCCAATC-3′
PI3K	Forward	5′-AGCATCCCCTCCGTGCCCAA-3′
	Reverse	5′-GAAGGCGGGGGAGGGGAGAG-3′
Akt	Forward	5′-ATGAACGACGTAGCCATTGTG-3′
	Reverse	5′-TTGTAGCCAATAAAGGTGCCAT-3′
mTOR	Forward	5′-TGGAGGTTACCGGTCTCGAT-3′
	Reverse	5′-AACAGGATGGTGGAGTGCTG-3′
*β*-Actin	Forward	5′-CCACCATGTACCCAGGCATT-3′
	Reverse	5′-CGGACTCATCGTACTCCTGC-3′

## Data Availability

The labeled dataset used to support the findings of this study are available from the corresponding author upon request.
